The article "Circ_0008068 facilitates the oral squamous cell carcinoma development by microRNA-153-3p/acylgycerol kinase (AGK) axis" was retracted in 2026. Reasons: concerns about the data; concerns about the results or conclusions.

# Circ_0008068 facilitates the oral squamous cell carcinoma development by microRNA-153-3p/acylgycerol kinase (AGK) axis

**DOI:** 10.1080/21655979.2022.2074106

**Published:** 2022-05-29

**Authors:** Yuanyuan Long, Chenxing Li, Baoyu Zhu

**Affiliations:** a Department of Prosthodontics, The First Affiliated Hospital of Zhengzhou University, Zhengzhou, Henan, China; b Department of Oral and Maxillofacial Surgery, Henan Provincial Stomatological Hospital, Zhengzhou, Henan, China; c Department of Oral and Maxillofacial Surgery, The First Affiliated Hospital of Zhengzhou University, Zhengzhou, Henan, China

**Keywords:** Oral squamous cell carcinoma, circ_0008068, miR-153-3p, AGK

## Abstract

Oral squamous cell carcinoma (OSCC) is a common cancer with high recurrence, metastasis rates and poor prognosis. Circular RNAs (circRNAs) take part in regulating OSCC. Herein, we examined the role of circ_0008068 in OSCC. The circ_0008068, Katanin p60 ATPase-containing subunit A-like 1 (KATNAL1) mRNA, microRNA-153-3p (miR-153-3p) and acylgycerol kinase (AGK) contents were indicated by quantitative real-time polymerase chain reaction (qRT-PCR) and western blot. Moreover, in vitro and in vivo assays were conducted to scrutinize the effects of circ_0008068 on OSCC. Additionally, the contact between miR-153-3p and circ_0008068 or AGK was assessed by dual-luciferase reporter assay and RNA immunoprecipitation (RIP) assay. Thereafter, we found that the appearance of circ_0008068 and AGK was increased, and miR-153-3p content was diminished in OSCC. Circ_0008068 lack subdued cell proliferation, migration, invasion, tube formation and glycolysis metabolism, but stimulated cell apoptosis in OSCC. In addition, circ_0008068 bound to miR-153-3p to modulate the expression of its target AGK. Besides, miR-153-3p was validated to act as a tumor suppressor in OSCC tumorigenesis by suppressing AGK. Additionally, circ_0008068 knockdown also attenuated tumor growth in nude mice. In all, circ_0008068 expedited the growth of OSCC by miR-153-3p/AGK axis.

**Abbreviations:** OSCC: Oral squamous cell carcinoma; AGK: Acylgycerol kinase; CircRNA: Circular RNA; KATNAL1: Katanin p60 ATPase-containing subunit A-like 1; qRT-PCR: Quantitative real-time polymerase chain reaction; miRNAs/miRs: MicroRNAs; RIP: RNA immunoprecipitation; 3′UTR3’: -untranslated region; HK2: Hexokinase 2; LDHA Lactate dehydrogenase A; IHC: Immunohistochemistry; CCK8: Cell counting kit-8; GAPDH: Glyceraldehyde-3-phosphate dehydrogenase

## Highlights

- Circ_0008068 silencing suppressed OSCC cell malignant phenotypes and glycolysis.
- Circ_0008068 acted a sponge for miR-153-3p to up-regulate its target AGK.
- Knockdown of circ_0008068 impeded OSCC growth in vivo.
- Circ_0008068 performed its oncogenic role via miR-153-3p/AGK axis.

The article "Circ_0008068 facilitates the oral squamous cell carcinoma development by microRNA-153-3p/acylgycerol kinase (AGK) axis" was retracted in 2026. Reasons: concerns about the data; concerns about the results or conclusions.

## 1. Introduction

Oral squamous cell carcinoma (OSCC) accounts for 95% of all head and neck cancers [1,2]. OSCC is highly metastatic, with a 5-year survival of less than 50% [3]. The prognosis for OSCC is poor. Despite great advances in treatment have been made, such as chemotherapy, in recent decades, therapeutic outcomes remain disappointing [4]. Hence, investigating the molecular mechanisms that regulate OSCC metastasis is critical for the development of specific diagnostic approaches and treatments.

Circular RNAs (circRNAs) belong to a kind of covalently closed looped RNAs that have no 5’-caps and 3’-tails, which can stabilize existence in plentiful types of organisms [5,6]. An increasing body of researches reveal that circRNAs have vital impacts on numerous cancers [7,8]. For example, hsa_circ_0001874 acted as a biomarker for the judgment of OSCC [9]. Circ_0000140 destroyed OSCC metastasis [10]. In addition, circ_100290 regulated OSCC cell growth and glycolysis [11]. Circ_002178 accelerated the proliferation of OSCC cells [12]. Besides, hsa_circ_0011946 facilitated cell invasion of OSCC [13]. Circ_0008068 is derived from the Katanin p60 ATPase-containing subunit A-like 1 (KATNAL1) gene (exons 2–9), it locates at chr13: 30,801,548–30,857,928 with the length of 11,615 bp. A recent study showed that circ_0008068 was upregulated in the saliva from the OSCC patients compared with the healthy controls [9]. However, the effects of circ_0008068 on OSCC are still not clear.

MicroRNAs (miRNAs/miRs) are a kind of RNA that ulteriorly adjust many cell developments [5,6]. For example, miR-133a-3p impeded OSCC cell invasion [14]. In addition, miR-31 regulated OSCC cell metastasis [10]. Moreover, miR-935 hindered OSCC progression [15]. Besides, miR-153-3p was found to regulate epithelial-mesenchymal transition (EMT) in OSCC cells [16,17]. Previous findings indicate that circRNAs can serve as ‘miRNA sponge’ and prevent miRNA-mediated degradation of mRNAs [18]. Preliminary bioinformatics analysis results reveled the binding sites of miR-153-3p and circ_0008068. It is indistinct whether circ_0008068 can regulate OSCC tumorigenesis via interacting with miR-153-3p. Acylgycerol kinase (AGK) is a lipid kinase that supports glycolytic metabolism [19]. The inhibition of AGK impaired tumor antigen-specific CD8^+^, which also suppressed CD8^+^ T cell growth [20]. AGK is vital for cell proliferation [21]. In addition, Liu *et al*. showed that AGK was highly expressed in OSCC and AGK knockdown suppressed OSCC cell proliferation and cell cycle progression [22]. Besides that, AGK acted as a target of miRNAs, including miR-610 and miR-194, to reverse the anticancer effects of them in OSCC [23,24]. All the findings indicated the implication of AGK in OSCC. Data of preliminary bioinformatics analysis showed that miR-153-3p could target AGK protein. However, the interaction of them in OSCC cells, as well as in the progression of OSCC, is still uncertain.

The article "Circ_0008068 facilitates the oral squamous cell carcinoma development by microRNA-153-3p/acylgycerol kinase (AGK) axis" was retracted in 2026. Reasons: concerns about the data; concerns about the results or conclusions.

In this work, we hypothesized that circ_0008068 might have functions in OSCC progression partially by regulating miR-153-3p and AGK. We exposed the role of circ_0008068 in OSCC cell growth, metastasis, and glycolysis and the underlying molecular mechanisms for the first time. The study disclosed that circ_0008068 expedited tumor growth by miR-153-3p/AGK axis. Our outcomes may be an advance for target therapy theory of OSCC.

## 2. Materials and methods

### 2.1 Clinical samples

The experiment was permitted by The First Affiliated Hospital of Zhengzhou University ((No.20192064). Thirty-seven pairs of OSCC tissues and corresponding normal tissues were collected from newly diagnosed OSCC patients with the signed informed consents. Details of volunteers are presented in Table 1.

**Table 1.** Associations between circ_0008068 expression and clinical features in OSCC patients (n = 37)

		Circ_0008068 expression (n)		
Clinical feature	Cases (n)	High [19]	Low [18]	*P*
**Age**				0.8859
≤60 years	21	11	10	
>60 years	16	8	8	
**Gender**				0.2536
Female	20	12	8	
Male	17	7	10	
**Lymph node metastasis**				0.0263*
Yes	25	16	9	
NO	12	3	9	
**TNM stage**				0.0035*
I–II	12	2	10	
III	25	17	8	
**Tumor size (cm)**				0.0016*
≤3	15	3	12	
>3	22	16	6	
**Histology grade**				0.0201*
Grade 1	15	4	11	
Grade 2 + 3	22	15	7	

^a^The median of relative circ_0008068 expression level is 2.14 so the number of high circ_0008068 expression is 19 (≥2.14)

### 2.2 Cell lines

The human OSCC cell lines CAL27, HSC-2 and SCC25, as well as normal HOK cells were obtained from American type culture collection (ATCC, Manassas, VA, USA) and cultivated in Dulbecco’s modified Eagle’s medium (DMEM, Invitrogen, Carlsbad, CA, USA) with 10% fetal bovine serum (FBS) in an environment with 5% CO_2_.

### 2.3 Quantitative real-time polymerase chain reaction (qRT-PCR) and RNA degradation assay

RNAs were prepared by Trizol (Takara, Tokyo, Japan) and were reverse-transcribed into complementary DNAs (cDNAs) with PrimeScript RT reagent Kit (Takara, Dalian, China). The SYBR Green kit (Takara) was conducted to carry out qRT-PCR. The glyceraldehyde-3-phosphate dehydrogenase (GAPDH) and U6 were used as controls. The gene contents were computed by the 2^−ΔΔCt^ method. RNase R treatment (Sigma-Aldrich, St. Louis, MO, USA) was conducted to confirm the cyclic form of circ_0008068. The primers as Table 2.

The article "Circ_0008068 facilitates the oral squamous cell carcinoma development by microRNA-153-3p/acylgycerol kinase (AGK) axis" was retracted in 2026. Reasons: concerns about the data; concerns about the results or conclusions.

**Table 2.** Primers for PCR

Name		Primers for PCR (5’-3’)
circ_0008068	Forward	TTCCCGTGGGACATTGATGA
	Reverse	AGTCGTAATTTCCAAGAAGGGCA
AGK	Forward	GCTTGACCCGACAAGCAAAG
	Reverse	ACGCAGCTTCACTATGTTCTCT
miR-153-3p	Forward	ACACTCCAGCTGGGTTGCATAGTCACAAA
	Reverse	CAGTGCGTGTCGTGGAGT
miR-140-5p	Forward	GCCGAGCAGTGGTTTTACCC
	Reverse	CAGTGCGTGTCGTGGAGT
miR-182-5p	Forward	GCCGAGTTTGGCAATGGTAGAA
	Reverse	CAGTGCGTGTCGTGGAGT
miR-197	Forward	GCCGAGTTCACCACCTTCTCCA
	Reverse	CAGTGCGTGTCGTGGAGT
miR-637	Forward	GCCGAGACTGGGGGCTTTCGGG
	Reverse	CAGTGCGTGTCGTGGAGT
miR-7	Forward	GCCGAGCAACAAATCACAGTCT
	Reverse	CAGTGCGTGTCGTGGAGT
GAPDH	Forward	TCCCATCACCATCTTCCAGG
	Reverse	GATGACCCTTTTGGCTCCC
U6	Forward	CTCGCTTCGGCAGCACATATACT
	Reverse	ACGCTTCACGAATTTGCGTGTC
KATNAL1	Forward	AAGGGAAGTGGAGGTCTCTGA
	Reverse	GAATCTGCTGCATCACCCCC

### 2.4 Western blot

The performance of western blot was conducted as some time ago published [25]. The antibodies were listed as follows: anti-AGK (ab137616; 1:500; Abcam, Cambridge, MA, USA), anti- Hexokinase 2 (HK2) (ab273721; 1:1,000; Abcam), anti-Lactate dehydrogenase A (LDHA) (ab101562; 1:500; Abcam).

### 2.5 Cell transfection

The small interfering RNA (siRNA) targeting back splice junction of circ_0008068 (si-circ_0008068, 5′-CCCAACAGGTCTCTGAAAGAAdtdt-3′) and the nontargeted siRNA (si-NC, 5′-TTCTCCGAACGTGTCACGT-3′) were by synthesized by Ribobio (Guangzhou, China). The short hairpin RNA (shRNA) was synthesized based on siRNA, then synthesized shRNA and the negative control were subcloned into the pLL3.7 vector (Geenseed, Guangzhou, China) to construct RNAi vector, named as sh-circ_0008068 (5′-CCGGCCCAACAGGTCTCTGAAAGAACTCGAGTTCTTTCAGAGACCTGTTGGGTTTTTG-3′) and sh-NC (5′-TTCTCCGAACGTGTCACGTTCA AGAGACGTGACACGTTCGGAGAATTTTTT-3′). MiR-153-3p mimics (miR-153-3p), miR-153-3p inhibitors (anti-miR-153-3p) and the controls (miR-NC or anit-miR-NC), as well as AGK overexpression plasmid (AGK) and the control plasmid (vector) were attained from Ribobio. Lipofectamine 2000 (Sigma) was conducted to execute the transient transfection. Lentiviruses carrying sh-circ_0008068 and sh-NC were purchased from Hanbio Biotechnology (Shanghai, China) for animal experiments.

### 2.6 Cell proliferation assay

CAL27 and SCC25 (2.0 × 10^3^/well) cells were planted in 96-well plates. Cell proliferation was detected at 0, 24, 48 and 72 h. In each well, 20 µL of Cell counting kit-8 (CCK-8) (Beyotime, Shanghai, China) solution (5 mg/mL) was supplemented. Then, the absorbance values at 450 nm were measured. Meanwhile, 5-Ethynyl-2’-deoxyuridine (EdU) assay with the Cell-Light™ EdU kit (Ribobio, China) was also utilized to assess cell proliferation as described before [26].

The article "Circ_0008068 facilitates the oral squamous cell carcinoma development by microRNA-153-3p/acylgycerol kinase (AGK) axis" was retracted in 2026. Reasons: concerns about the data; concerns about the results or conclusions.

### 2.7 Transwell assay

The migration of CAL27 and SCC25 cells was assessed by a transwell with 8 μm pore polycarbonate membrane (BD Biosciences, Bedford, MA, USA). In brief, 4 × 10^5^ transfected OSCC cells, resuspended in 100 µL DMEM without serum, were planted into the upper chamber. Then, the lower chamber of the transwell was added with 500 µL of DMEM and 10% FBS. The same method was enforced to detect the invasion ability, but the transwell chamber were pre-coated with matrigel (BD Biosciences). Eventually, a light microscope was used to determine the count of cells.

### 2.8 RNA immunoprecipitation (RIP) assay

The Magna RIP kit (Sigma) was utilized to carry out the RIP assay along with the specification [27]. CAL27 and SCC25 cells were lysed with RIP buffer, cell lysates were then incubated with the magnetic beads and anti-Ago2 or anti-IgG at 4°C overnight. Later on, the immunoprecipitated RNA was isolated for qRT-PCR.

### 2.9 Matrigel tube formation assay

A 96-well plate was pre-coated with Matrigel and allowed to polymerize for 30 min at 37°C. The conditioned medium of CAL27 and SCC25 cells with assigned transfection was collected. Thereafter, HUVECs with conditioned medium were seeded onto matrigel plates at 2.5 × 10^4^ cells/well and incubated for 24 h. ImageJ software (NIH, Bethesda, MD, USA) was used to observe the number of tubes and branches. The elongated multi-cellular structures were considered as tube-like structures. The intersecting points of two or more tubes were considered as branches.

### 2.10 Flow cytometry assay

OSCC cells were seeded into 6-well plates. As the defined by Wang *et al*., the Annexin V-FITC/PI kit (Sigma) was engaged [28]. Finally, a BD FACSCalibur™ flow cytometry (BD Biosciences) was applied to evaluate the count of apoptotic cells.

### 2.11 Dual-luciferase reporter assay

The direct relations between miR-153-3p and circ_0008068 or AGK 3’ untranslated region (3ʹUTR) were estimated by starbase. The circ_0008068 and AGK wild (WT) and mutant (MUT) sequences produced by Ribobio were inserted into the pmirGLO luciferase vectors to establish luciferase reporter vectors (WT-circ_0008068, WT-AGK 3ʹUTR or MUT-circ_0008068, MUT-AGK 3ʹUTR). The recombinant vectors were cotransfected into OSCC cells with miR-NC or miR-153-3p. Finally, the luciferase activity was scrutinized.

### 2.12 Xenograft models

The experiments abided the supervision of the Animal Care and Use Committee of The First Affiliated Hospital of Zhengzhou University. The nude mice were gotten from Shanghai Laboratory Animal Company (SLAC, Shanghai, China). CAL27 cells (5 × 10^6^) with sh-circ_0008068 or the sh-NC were vaccinated into mice (n = 6/group; 6 weeks; female; 18–22 g). The tumor volume was assessed as the formula: volume = length × width^2^ × 0.5. Four weeks later, the tumor tissues were engraved for next investigation. All animal experiments were approved by the Animal Care and Use Committee of The First Affiliated Hospital of Zhengzhou University and complied with the guidelines of the National Institutes of Health.

The article "Circ_0008068 facilitates the oral squamous cell carcinoma development by microRNA-153-3p/acylgycerol kinase (AGK) axis" was retracted in 2026. Reasons: concerns about the data; concerns about the results or conclusions.

### 2.13 Immunohistochemistry (IHC) assay

The Ki67 (ab92742; 1:1,000; Abcam) abundance in tumors was distinguished by IHC assay. The explicit examination mode was in keeping with the explanation of Ma *et al*. [29]. In the end, the slides were perceived.

### 2.14 Statistical assay

Data are manifested as mean ± standard deviation (SD). All experiments were repeated three times. The correlation between groups was analyzed by Pearson correlation analysis. The difference was evaluated by the Student’s *t*-test and analysis of variance (ANOVA) with hoc post Turkey test in SPSS 23.0. *P* < 0.05 was significant.

## 3. Results

We hypothesized that circ_0008068 might have functions in OSCC progression partially by regulating miR-153-3p and AGK. This study aimed to investigate the role of circ_0008068 in OSCC cell growth, metastasis, and glycolysis and the underlying molecular mechanisms for the first time. Through the in vitro and in vivo assays, we disclosed that circ_0008068 expedited tumor growth by miR-153-3p/AGK axis.

### 3.1 Circ_0008068 was elevated in OSCC tissues and cells

Initially, circ_0008068 expression was higher in OSCC tumor tissues (Figure 1(a)). Besides, the correlation between circ_0008068 expression and clinical characteristics in OSCC patients was showed in Table 1. The expression of circ_0008068 was significantly correlated with lymph node metastasis, TNM stage and tumor size (cm) (Figure 1(b) and Table 1) (P < 0.05). Table 1 also shows that the expression of circ_0008068 was significantly correlated with histology grade (P = 0.0201). Besides, the appearance of circ_0008068 was higher in the low-overall survival group (Fig. S1). In addition, the circ_0008068 contents were notably higher in OSCC cells (CAL27, HSC-2 and SCC25) than control cells (HOK) (Figure 1(c)). Because the circ_0008068 content was much higher in CAL27 and SCC25 cells, these two types of cells were selected for subsequent tests. As shown in Figure 1(d), circ_0008068 is located in chr13:30801548–30857928 and the structure was circular RNAs. In addition to this, to further confirm the structure of circ_0008068, an RNase R enzyme (a highly processive 3’ to 5’ exoribonuclease) assay was enforced to distinguish the structure of circ_0008068 and KATNAL1 mRNA in CAL27 and SCC25 cell lines. As displayed in Figure 1(e,f), KATNAL1 mRNA was observably reduced after RNase R treatment when compared with the circ_0008068. The result further confirmed the cyclic form of circ_0008068. These consequences discovered that circ_0008068 was elevated in OSCC.

The article "Circ_0008068 facilitates the oral squamous cell carcinoma development by microRNA-153-3p/acylgycerol kinase (AGK) axis" was retracted in 2026. Reasons: concerns about the data; concerns about the results or conclusions.

**Figure 1.** Circ_0008068 appearance was enhanced in OSCC.

(a and b) The expression of circ_0008068 in OSCC tissues (n = 37) and paracancer tissues (n = 37) was detected by qRT-PCR. (c) The expression of circ_0008068 in HOK, CAL27, HSC-2 and SCC25 cells was examined by qRT-PCR (n = 3). (d) The structure of circ_0008068. (e and f) The relative levels of circ_0008068 and KATNAL1 mRNA were determined after treatment with RNase R by qRT-PCR (n = 3). *P < 0.05.

### 3.2 Circ_0008068 lack restrained OSCC cell tumorigenesis

The circ_0008068 content was delimited in OSCC cells by si-circ_0008068 (Figure 2(a,b)). Besides, circ_0008068 lack reduced cell proliferation (Figure 2(c–e)). Afterward, the knockdown of circ_0008068 repressed the migration and invasion of CAL27 and SCC25 cells (figure 2(f,g)). Additionally, circ_0008068 absence subdued tube formation of vascular endothelial cells (Figure 2(h)). Besides, circ_0008068 downregulation encouraged cell apoptosis in OSCC cells (Figure 2(i)). Then, the knockdown of circ_0008068 significantly repressed glycolysis metabolism in OSCC cells (Figure 2(j,k)). HK2 and LDHA were linked with glycolysis metabolism. We certified that si-circ_0008068 abridged the levels of HK2 and LDHA in OSCC cells (Figure 2(l)).

**Figure 2.** Circ_0008068 lack subdued OSCC tumorigenesis.

(a–l) OSCC cells were transfected with si-NC or si-circ_0008068. (a and b) The circ_0008068 content was quantified. (c and d) The impact of circ_0008068 deletion on the viability of OSCC cells was illustrated by CCK8 assay. (e) The cell proliferation was measured by EdU assay. Scale bar, 100 μm. (f and g) The influence of circNFATC3 deletion on cell migrated and invasion was measured. Scale bar, 50 μm. (h) The number of branches was detected. Scale bar, 50 μm. (i) The impact of circ_0008068 knockdown on apoptosis of CAL27 and SCC25 cells. (j and k) The glycolysis metabolism were examined. (l) The HK2 and LDHA contents were examined. n = 3, *P < 0.05.

### 3.3 MiR-153-3p was targeted by circ_0008068 in OSCC cells

As shown in Figures 3(a,b), the RNA samples from the cytoplasm and the nuclear of CAL27 and SCC25 cells were extracted respectively, and circ_0008068 was mostly disseminated in the cytoplasm relative to the nucleus. Starbase was implemented to foresee the miRNAs that might be interacted with circ_0008068, among which, miR-140-5p, miR-153-3p, miR-182-5p, miR-197, miR-637, and miR-7 were found to be deregulated in OSCC according to previous findings. After si-circ_0008068 transfection, the alteration of miR-153-3p content was the most obvious, so it was selected as a further experimental target (Fig. S2A and B). The targeted binding site was showed (Figure 3(c)). The miR-153-3p level was augmented by miR-153-3p mimic (Figure 3(d)). The decreased luciferase activity in OSCC cells transfected with WT-circ_0008068 and miR-153-3p was validated using the dual-luciferase reporter assay (Figure 3(e,f)). It has been widely known that miRNAs regulate target gene expression by binding to Argonaute 2 (AGO2), the key component of RNA-induced silencing complex (RISC). Then RIP assay was conducted, results certified that miR-153-3p and circ_0008068 in CAL27 and SCC25 cells were efficiently pulled down by anti-Ago2 antibodies compared with IgG (Figure 3(g,h)), further indicating the binding between miR-153-3p and circ_0008068. Thereafter, the data demonstrated that miR-153-3p level was diminished in OSCC tissues (Figure 3(i)), which was negatively correlated with circ_0008068 expression (Figure 3j). Meanwhile, a decreased miR-153-3p was also observed in OSCC cells (Figure 3(k)). The appearance of miR-153-3p was declined by anti-miR-153-3p (Figure 3(l)). Besides, the appearance of miR-153-3p was augmented by si-circ_0008068, whereas was diminished by anti-miR-153-3p (Figure 3(m,n)).

The article "Circ_0008068 facilitates the oral squamous cell carcinoma development by microRNA-153-3p/acylgycerol kinase (AGK) axis" was retracted in 2026. Reasons: concerns about the data; concerns about the results or conclusions.

**Figure 3.** Circ_0008068 acted as a sponge for miR-153-3p.

(a and b) The circ_0008068 appearance was quantified. (c) The binding sites of circ_0008068 and miRNAs was forecast by Starbase. (d) The efficiency of miR-153-3p mimic was evaluated (n = 3). (e–h) The association of circ_0008068 and miR-153-3p by dual-luciferase reporter assay and RIP assay (n = 3). (i) The appearance of miR-153-3p in OSCC tissues was detected (n = 37). (j) MiR-153-3p expression was negatively correlated with circ_0008068 expression in OSCC tissues. (k) The appearance of miR-153-3p in OSCC cells was detected (n = 3). (l) The knockdown efficiency of anti-miR-153-3p or anti-miR-NC (n = 3). (m and n) The appearance of miR-153-3p was detected in OSCC cells co-transfected with si-circ_0008068 and anti-miR-153-3p (n = 3).*P < 0.05.

### 3.4 Circ_0008068 expedited OSCC via miR-153-3p

To further research the influences between circ_0008068 and miR-153-3p on OSCC progression, we discovered that circ_0008068 knockdown decreased cell proliferation in CAL27 and SCC25 cells, while this consequence was lessened by anti-miR-153-3p (Figure 4(a-c)). Moreover, transwell assay demonstrated that anti-miR-153-3p attenuated the destruction influences of circ_0008068 lack on cell migration and invasion in OSCC cells (Figure 4(d,e)). Furthermore, the downregulation of circ_0008068 inhibited tube formation of vascular endothelial cells, whereas miR-153-3p inhibitor lessened the impact (figure 4(f)). On the other hand, flow cytometry analysis indicated that in CAL27 and SCC25 cells, anti-miR-153-3p incompletely restored the advancement effect of circ_0008068 lack on apoptosis (Figure 4(g)). Afterward, circ_0008068 absence repressed glycolysis metabolism in OSCC cells, but this impact was partially attenuated by anti-miR-153-3p (Figure 4(h,i)). The anti-miR-153-3p lessened the influences of circ_0008068 lack on the declined HK2 and LDHA contents in OSCC cells (Figure 4j).

The article "Circ_0008068 facilitates the oral squamous cell carcinoma development by microRNA-153-3p/acylgycerol kinase (AGK) axis" was retracted in 2026. Reasons: concerns about the data; concerns about the results or conclusions.

**Figure 4.** Circ_0008068 assisted OSCC via miR-153-3p.

(a–j) OSCC cells were co-transfected with si-circ_0008068 and anti-miR-153-3p. (a–c) The cell proliferation, (d) migration, (e) invasion, (f) the number of branches, (g) cell apoptosis, (H and I) the glycolysis metabolism, (j) as well as levels of HK2 and LDHA were inspected. n = 3, *P < 0.05.

### 3.5 MiR-153-3p targeted AGK in CAL27 and SCC25 cells

The miR-153-3p was forecasted including the binding sites of AGK 3ʹUTR (Figure 5(a)). The luciferase activity of WT-AGK 3ʹUTR was abridged by miR-153-3p, but in the MUT-AGK 3ʹUTR group luciferase activity was not expressively altered (Figure 5(b,c)). RIP assay upshots certified the contact of miR-153-3p and AGK in OSCC cells (Figure 5(d,e)). Consequences presented that AGK levels were upregulated in OSCC cells and tumor tissues (figure 5(f–h)). Besides that, AGK expression level in OSCC tissues was negatively correlated with miR-153-3p expression (Figure 5(i)), and positively correlated with circ_0008068 expression (Figure 5(j)). After the AGK transfection, the AGK expression was augmented compared with the vector group (Figure 5(k)). Moreover, AGK reserved the inhibition influences of miR-153-3p on the appearance of AGK in CAL27 and SCC25 cells (Figure 5 ()l).

**Figure 5.** MiR-153-3p targeted AGK in CAL27 and SCC25 cells.

(a) The binding sites between miR-153-3p and AGK was scrutinized. (b-e) The connection between miR-153-3p and AGK dual-luciferase reporter assay and RIP assay (n = 3). (f–h) The appearance of AGK was detected in OSCC tissues (n = 37) and cells (n = 3). (i, j) AGK expression was negatively correlated with miR-153-3p expression, and positively c correlated with circ_0008068 expression in OSCC tissues. (k) The transfection efficiency of AGK or vector in OSCC cells (n = 3). (l) The appearance of AGK was detected in OSCC cells co-transfected with miR-153-3p and AGK (n = 3). *P < 0.05.

### 3.6 MiR-153-3p repressed OSCC by AGK

The miR-153-3p abridged the cell proliferation of OSCC cells, while this impact was restricted by AGK overexpression (Figure 6(a–c)). Subsequently, the migration and invasion of CAL27 and SCC25 cells were suppressed by miR-153-3p mimic, however, AGK could partially abolish these impacts (Figure 6(d,e)). Furthermore, AGK lessened the inhibition influences of miR-153-3p on tube formation of vascular endothelial cell (figure 6f). In flow cytometry analysis, we confirmed that miR-153-3p mimic expedited the apoptosis of CAL27 and SCC25 cells, and this influence was delimited by AGK (Figure 6(g)). Afterward, the miR-153-3p mimic significantly repressed glycolysis metabolism in OSCC cells, but this influence was incompletely weakened by AGK (Figure 6(h,i)). The HK2 and LDHA contents in CAL27 and SCC25 cells were moderated by miR-153-3p mimic, whereas AGK diminished the impacts (Figure 6(j)). Furthermore, AGK expression dwindled by si-circ_0008068 in OSCC cells, which was partially rescued by anti-miR-153-3p introduction (Figure 7(a–d)).

The article "Circ_0008068 facilitates the oral squamous cell carcinoma development by microRNA-153-3p/acylgycerol kinase (AGK) axis" was retracted in 2026. Reasons: concerns about the data; concerns about the results or conclusions.

**Figure 6.** MiR-153-3p suppressed OSCC progression via AGK.

(a–j) OSCC cells were co-transfected with miR-153-3p and AGK. (a–c) The cell proliferation, (d) migration, (e) invasion, (f) the number of branches, (g) cell apoptosis, (h and i) the glycolysis metabolism, (j) and the HK2 and LDHA contents were inspected. n = 3, *P < 0.05.

**Figure 7.** The appearance of AGK in OSCC cells.

(a–d) The appearance of AGK was measured by qRT-PCR and western blot in OSCC cells co-transfected with si-circ_0008068 and anti-miR-153-3p. n = 3, *P < 0.05.

### 3.7 Circ_0008068 lack limited tumor growth

The CAL27 cells infected with lentivirus carrying sh-circ_0008068 or sh-NC were vaccinated into athymic nude mice to conduct in vivo assay. As shown in Figure 8(a–c), we found that intratumoral injection of sh-circ_0008068 reserved tumor volume and weight. Additionally, the appearance of circ_0008068 and AGK was abridged, while the miR-153-3p content was augmented in the sh-circ_0008068 group (Figure 8(d,e)). Thereafter, HE pathological sections of the tumors were shown, and the down-regulation of circ_0008068 could remarkably suppress tumor growth (figure 8f). Besides that, the Ki67 content was lesser in the sh-circ_0008068 group, designating that circ_0008068 lack repressed tumor growth (figure 8(f)). These consequences designated that circ_0008068 lack subdued tumor growth *in vivo* via miR-153-3p/AGK axis.

**Figure 8.** Circ_0008068 lack delimited tumor growth by suppressing AGK via miR-153-3p.

(a-c) Tumor volumes and weight was observed. (d and e) The appearance of circ_0008068, miR-153-3p and AGK was detected by qRT-PCR and western blot. (f) HE staining of tumors was showed, and IHC assay was accomplished to assess the appearance of Ki67 in the tumors. Scale bar, 50 μm. n = 6, *P < 0.05.

The article "Circ_0008068 facilitates the oral squamous cell carcinoma development by microRNA-153-3p/acylgycerol kinase (AGK) axis" was retracted in 2026. Reasons: concerns about the data; concerns about the results or conclusions.

## 4. Discussion

The occurrence of metastases acts as a key part in the treatment of OSCC, with lung metastases accounting for approximately 70% of cases [30]. Therefore, detailed research of the molecular underlying long-distance metastasis may facilitate the advance of analytic for OSCC. Previous sequencing consequences exhibited that there were numerous differentially circRNAs in OSCC tissues. Some emerging circRNAs acted crucial characters in OSCC progression. For instance, circRNA mitochondrial translation optimization 1 homologue promoted OSCC cell proliferation, migration, and invasion *in vitro* via miR-320a/alpha thalassemia/mental retardation, X-linked (ATRX) axis [31]. Circ_0005320 silencing impeded OSCC growth *in vivo* and *in vitro* by sponging miR-486-3p and miR-637 [32]. Besides, hsa_circ_100533 could prevent OSCC [33]. Compare with previous findings, we firstly confirmed that circ_0008068 facilitated OSCC development by regulating cancer cells proliferation, invasion, migration. Moreover, we also demonstrated that circ_0008068 silencing could suppress glycolysis, a glycometabolism that was preferentially adopted by cancer cells to produce more energy for their sustaining growth [34], by decreasing glycolytic enzyme HK2 and lactate production in OSCC cells. Importantly, our animal study further discovered that circ_0008068 lack impaired tumor evolution. CircRNAs could bind to miRNAs, like circ_100290 targeted miR-29 family and circ_100533 regulated miR-933 in OSCC [33,35]. Here, we verified that circ_0008068 directly targeted miR-153-3p, and enhanced OSCC progression by adjusting miR-153-3p.

MiR-153-3p was revealed to perform anticancer effects in the advancement of malignant melanoma, acute lymphoblastic leukemia and breast cancer [36–38]. Herein, we established the suppression role of miR-153-3p in OSCC tumorigenesis. Previous evidence has illustrated that circRNA-miRNA-mRNA network was involved in the progression of OSCC [39]. Thus, the underlying mRNAs of miR-153-3p was investigated, and we found that miR-153-3p targeted AGK. The formerly described that AGK could target T cell membrane to regulate the anti-tumor immunity of cells. Meanwhile, AGK could enhance glycolysis to facilitate the CD8^+^ T cell response. In light of previous studies, the study of AGK has led to a deeper comprehension of the interactions between cell signaling and metabolic rate, and has opened up new therapeutic pathways for targeting cancer and immune-mediated diseases [20]. In this paper, the expression of AGK was improved in OSCC. The miR-153-3p increase subdued cell growth, metastasis and glycolysis, and these influences were diminished by AGK. In addition, miR-153-3p lack suppressed the impact of circ_0008068 silencing on AGK content in OSCC cells, further revealing the circ_0008068/miR-153-3p/AGK axis in OSCC tumorigenesis. This paper has some significant findings; however, it still has some limitations. For example, the results obtained from commercial cell lines are not completely representative of the actual conditions *in vivo*. The results of this study are not supported by clinical trial data. We will implement the experiment to indicate the character of circ_0008068 in clinical application.

The article "Circ_0008068 facilitates the oral squamous cell carcinoma development by microRNA-153-3p/acylgycerol kinase (AGK) axis" was retracted in 2026. Reasons: concerns about the data; concerns about the results or conclusions.

## 5. In conclusion

Herein, the paper revealed that circ_0008068 and AGK were abundantly expressed and miR-153-3p was poor expressed in OSCC. Additionally, our paper manifested that circ_0008068 knockdown repressed OSCC cell proliferation, migration, invasion, tube formation and glycolysis metabolism via miR-153-3p/AGK axis. This information could make available in the development of new therapy for OSCC handling.

## Supplementary Material

Supplemental Material

## Data Availability

Please contact the correspondence author for the data request.
